# Drug Resistance Mechanism of Enterobacteriaceae with Decreased Antibiotic Sensitivity

This article has been retracted.

**DOI:** 10.1155/2022/8285437

**Published:** 2022-10-10

**Authors:** Fang Rong, Yuanyuan Sun, Xiao Li, Chenhao Zhang

**Affiliations:** ^1^Wangjing Hospital, China Academy of Chinese Medical Sciences, Beijing 100102, China; ^2^Peking University People's Hospital, Beijing 100102, China; ^3^Yuxi People's Hospital, Yuxi, Yunan 653100, China

## Abstract

To investigate the mechanism of antibiotic resistance in Enterobacteriaceae. Carbapenem Enterobacteriaceae bacteria isolated from a hospital from January 2015 to June 2020 were selected. Drug resistance phenotype test, drug sensitivity test, and conjugation test were used to observe the drug sensitivity results and the titer of acrB antibody. Finally, the data were statistically analyzed. All strains were resistant to ceftazidime, ceftriaxone, ertapenem, and aztreonam. 87.5% of the samples were resistant to piperacillin. Multisite sequence typing showed that 5 carbapenem-resistant *Klebsiella pneumoniae* belonged to 4 different types. The sequence types of kpn6099 and kpn6617 were the same. In the sensitivity comparison, *Escherichia coli* J53 was more sensitive to these two antibiotics, minimum inhibitory concentration values were 0.5 and 0.25 *μ*g/ml, respectively. In addition, the sensitivity of *E. coli* J53 to carbapenems was slightly higher than that of kpn6617. The results showed that the enzyme-linked immunosorbent assay titer of acrB antibody was 1:40,000, and the preparation of acrB antibody was successful. Plasmid-mediated deletion of IMP-1 metallo-*β*-lactamase binding outer membrane protein is one of the main reasons for the decrease of antibiotic sensitivity.

## 1. Research Background

Once drug resistance occurs, the chemotherapeutic effect of the drug is significantly reduced. Drug resistance can be divided into acquired drug resistance and natural drug resistance according to its causes. Pathogens in nature, such as a strain of bacteria, may also have natural resistance. The characteristics of bacterial resistance is a major problem in the treatment of infectious diseases [1]. Bacteria can be resistant to a certain class of antibiotics, or to a variety of antibiotics with different chemical structures [2, 3]. According to the bacterial resistance, it can be divided into single drug resistance and multidrug resistance [4–6]. The former refers to the bacterial resistance to a certain class of antibiotics, which is caused by a single drug resistance factor; the latter refers to the bacterial resistance to multiple antibiotics mediated by chromosome and plasmid [7, 8]. The former does not depend on antibiotics, but is closely related to the heredity and evolution of bacteria. The latter is the result of gene mutation under selective pressure such as antibiotics, and is also related to the transfer and transmission of drug-resistant plasmids, transposons and integrons [9, 10].

For example, compared with foreign countries, the broad-spectrum polylactase producing *Escherichia coli* is more resistant to aminoglycosides, sulfonamides, and quinolones. *E. coli* isolated from urinary tract infection has a complex drug resistance mechanism. Most of the drug-resistant genes exist in plasmids, which are easy to cause the spread of drug resistance. This brings a lot of difficulties to the treatment. These pathogenic genes are usually encoded in mobile protoplasts and spread between different strains [11].

Generally speaking, bacterial resistance is mainly through the following mechanisms: the production of inactivated enzymes, resulting in the loss of drug activity or structural changes; changes in the permeability of bacterial cell membrane, so that drugs or disinfectants, detergents, and other chemicals cannot enter the bacteria; the target structure or quantity of antibacterial drugs changes, unable to effectively combine with antibacterial drugs; drugs are pumped out of the body through active efflux system, the drug cannot reach the threshold concentration of killing bacteria [12, 13].

Antibiotics are a class of secondary metabolites with anti-pathogen or other activities produced by microorganisms or higher animals and plants in the process of life, which can interfere with the developmental functions of other living cells. Usually, the above mechanisms occur simultaneously, which determines the resistance of some bacteria to certain antibiotics. According to the mechanism of action, active jet system can be divided into five superfamilies: ABC binding box superfamily, mainly promoting subfamilies and the drug-resistant nodal cell differentiation family. Except these, the others are energy dependent. Bacterial efflux pump system is mainly composed of transporters, additional proteins, and outer membrane proteins. The transporter is located on the cytoplasmic membrane and acts as a pump. The additional protein acts as a bridge between the outer membrane protein and the transporter. Outer membrane proteins are similar to channel proteins and are located in the cell wall or outer membrane [14]. These three proteins are indispensable to maintain the normal function of bacterial efflux system. Bacteria also have an active pump system, which excretes not only secondary metabolites, but also antibiotics [15].

## 2. Theoretical Basis

### 2.1. Enterobacteriaceae

Enterobacteriaceae bacteria are widely distributed and have a large host range. Humans, animals, and plants have parasitic or symbiotic, epiphytic, saprophytic, and can also survive in soil or water, and are closely related to humans. Enterobacteriaceae bacteria can cross-infect and spread between medical staff and patients, and also their genetic materials (such as plasmids or transposons) can be obtained from the outside world, leading to horizontal transmission of drug-resistant genes, which further leads to the wide spread of drug-resistant bacteria [16, 17]. In recent years, with the wide use of *β*-lactamases (ESBLs) and AmpC enzymes, ESBLs in Enterobacteriaceae can eliminate almost all cephalosporins except carbapenem, which makes carbapenem become an important substance in the treatment of clinical negative bacterial infections, and carbapenem-resistant Enterobacteriaceae has increased year-by-year [18, 19]. AmpC enzymes can be divided into three types according to their production patterns: induced high-yield enzymes, sustained high-yield enzymes, and sustained low-yield enzymes. The synthesis of high-yield enzymes is usually related to *β*-lactam antibiotics. Whether the enzyme is in the presence of *β*-lactam antibiotics or not, there is a high level of AmpC enzyme. The reason is that in order to prevent the mutation and regulate the mutation of ampD gene, one of the defective ampD proteins is produced. Because it does not form a protein complex with another regulatory protein ampr, it leads to the activation of ampr protein and the expression of AmpC enzyme is limited. With the wide application of *β*-lactam antibiotics, especially cephalosporins, the number of AmpC enzymes produced by Gram-negative bacteria is increasing, especially the emergence of AmpC enzyme and plasmid-mediated AmpC enzyme, which leads to the wide spread of drug-resistant strains. The resistance of Enterobacteriaceae to carbapenems is mainly caused by three mechanisms: first, the production of carbapenemases; second, the loss or down regulation of high-yield ESBLs or AmpC enzyme binding stomatal proteins, resulting in the decrease of sensitivity to carbapenems; third, the alteration of penicillin-binding protein (PBP), the target of carbapenems [20, 21]. *Klebsiella pneumoniae* carbapenemase (KPC) enzymes refer to carbapenemases produced in *K. pneumoniae*. One of the Enterobacteriaceae bacteria is *K. pneumoniae*. *K. pneumoniae* st258 carries KPC enzyme and is widely spread in the world, and *K. pneumoniae* st11 is the main type in China [22]. The main multisite sequence typing (MLST) typing of *K. pneumoniae* carrying KPC enzyme in China is consistent with the international MLST classification, which is ST131, and the mode of transmission is more complex and diverse [23]. Drug-resistant genes are located in the common region of plasmid, integron, transposon, or insertion sequence, and can be transferred horizontally, and horizontally spread in the same or different strains through coupling, transformation, transduction, and transposition [24, 25].

KPC enzyme can hydrolyze not only carbapenems, but also penicillins, cephalosporins, and aminoaspergillins [26]. New Delhi metallo-beta lactamase (NDM) is a common carbapenemase and belongs to type B according to Ambler classification. EDTA generally refers to ethylenediaminetetraacetic acid. EDTA is an organic compound whose chemical formula is C10H16N2O8. EDTA can inhibit the hydrolysis activity of these enzymes. Like KPC enzymes, class B enzymes are not currently inhibited by commercial lactam resistant inhibitors. Imipenemase metallo-*β*-lactamase (IMP) enzyme is a very common class B enzyme, which is the most common in *P. aeruginosa*. However, in recent years, the isolation rate of IMP enzyme in Enterobacteriaceae is also on the rise. The genetic environment of IMP enzymes is often complex and diverse, but it usually exists in integrons, and integrons can capture other gene cassettes. When integrons are associated with transposons or plasmids, IMP enzymes can also capture other gene cassettes, and stable transfer can be seen in a variety of bacteria. *E. coli* is a normal colonization bacterium in human body and one of the common conditional pathogens, can cause respiratory tract, urinary tract infection, and bacteremia. At present, *E. coli* is one of the normal colonization bacteria, and is also a common conditional pathogen. Although the incidence of clinical infection is lower than that of *K. pneumoniae*, it plays an important role in hospital and community-acquired infection. If we do not pay attention to the drug resistance research and take timely shielding measures, once it spreads among the population, the consequences will be unimaginable. They may be related to epidemiology. In particular, E2 and E4 belong to intensive care unit (ICU) and have the same MLST and pulsed-field gel electrophoresis typing. The drug resistance gene is carried by the 160 kb combined incfII plasmid. The two strains are transmitted through cloning and lead to infection of different patients in the same ward [27].

After multistage screening, a mutant strain T-E5 with stable characters and stronger activity was obtained. Strains E5 and E7 were from respiratory department and general surgery department, respectively, and had high genetic correlation. Nosocomial infection control is very important to slow down the spread of drug-resistant bacteria in hospitals. From the origin of drug resistance, inherent drug resistance is drug resistance does not depend on the existence of antibiotics, it has a greater relationship with heredity and evolution, and internal drug resistance is the stable genetic characteristics of bacteria itself, bacterial chromosome is controlled by DNA, which is the common characteristics of similar bacteria. Acquired drug resistance is caused by gene mutation or the transfer of mobile resistance factors under antibiotic pressure. The migration factors include plasmids, transposons, and integrons [28].

### 2.2. Antibiotic Sensitivity

Under the pressure of antibiotic selection, pathogens gradually form drug resistance, and infectious pathogens begin to produce drug resistance. The sensitivity was further reduced. More importantly, due to the irrational use of antibiotics, many pathogens have developed multidrug resistance. For example, compared with imipenem and meropenem, ertapenem may be more sensitive to the changes of outer membrane proteins and more suitable to indicate the changes of bacterial outer membrane proteins. Urinary tract infection refers to a large number of bacteria into the urinary tract, causing urinary tract inflammation. Urinary tract infection is one of the most common bacterial infections. At present, the diagnosis of chronic pyelonephritis should have the typical imaging manifestations of chronic pyelonephritis diagnosed by intravenous pyelography. Urinary tract infection can occur in any age group. At present, there are many kinds of antibiotics to treat urinary tract infection. The antibiotics used in urinary tract infection mainly include lactic acid lactam antibiotics and nitrofurantoin. Fluoroquinolones can replace sulfonamides and can be used as the first choice of drugs for urinary tract infection. Due to the rapid increase of drug resistance in vivo and the low resistance rate of other antibiotics, lactam antibiotics are not recommended as the first choice for empirical treatment of urinary tract infection.

At the same time of transmission, the original gene can obtain a new pathogenic gene; or it was previously encoded in a mobile plasma but inserted into the chromosome after mutation [29]. Urinary bacterial infection is a common infectious disease, mainly including asymptomatic bacteriuria, cystitis, and pyelonephritis. Pyelonephritis can endanger the life safety of patients. Molecular typing mainly includes multisite sequencing, ribosomal typing, and polymerase chain reaction (PCR) typing. The first two methods are time-consuming and laborious, while PCR typing can quickly and accurately cluster UPEC. According to PCR typing, *E. coli* can be divided into four types: A, BL, B2, and D. Type B2 is the most common type of urinary tract infection, followed by type D, while type A and BL are mainly intestinal symbionts. The main biological function of CNF-1 on HeLa cells is to make HeLa cells widely multinucleated and round, but cannot induce HeLa cells apoptosis. This cell line does not die from aging and can divide indefinitely. HeLa cells are usually used as cell models for *E. coli* adhesion tests [30]. Acquired drug resistance mainly includes resistance caused by gene mutation caused by mobile factors and resistance caused by antibiotic pressure. The change of outer membrane permeability: reduce the number of antibiotics entering bacteria and reduce the drug resistance of *E. coli* caused by antibiotics intake.

The overexpression of AcrAB–TolC efflux pump is one of the main mechanisms of multidrug resistance of Enterobacteriaceae, which is mainly composed of periplasmic fusion protein AcrA, outer membrane channel protein TolC, and drug proton transporter AcrB. Under normal circumstances, the normal expression of acrabtolc contributes to the resistance of *E. coli* to intestinal bile salts and other hydrophobic substances; however, its overexpression will lead to extensive drug resistance, including lactam, fluoroquinolones, tetracyclines, chloramphenicol, erythromycin, neomycin, and rifampicin. If inactivated, the sensitivity of the system to different types of antibiotics will be significantly increased. Overexpression of *P. aeruginosa* can significantly reduce the sensitivity of macrolides, aminoglycosides, and tetracyclines. Compared with the former, the latter is easier to spread in the environment. Drug-resistant plasmids are widely found in Gram-negative bacteria and Gram-positive bacteria. Drug-resistant plasmids are composed of two parts: the determinants of drug resistance and the transmission factors of drug resistance. These two parts can exist independently or as a whole, but there is no conjugate transfer when they exist alone. They are typical fungicides during the breeding season.

### 2.3. Drug Resistance Mechanism

At present, bacteria are known to be resistant to lactam antibiotics through the following three mechanisms: the production of inactivated enzymes. According to Bush classification and Ambler molecular classification, they were divided into four groups. The coding gene family includes CTX-M, OXA, SHV, GES/IBC, and so on. Metal caprolactam enzyme: metal ions as the active center. The main coding genes are IMP and VIM gene family. Except for lactamase inhibitors, there was no or only weak antibacterial activity. When combined with other lactam resistant antibiotics, it can significantly improve the antibacterial activity against penicillins and cephalosporins with unstable lactamase resistance. Different lactam antibiotics have different binding strength and quantity to PBPs, so different lactam antibiotics have different antibacterial effects. Therefore, the activities of these jet pumps may affect the invasion factors.

Gram-negative bacteria generally refers to bacteria that are red in the Gram staining reaction. In the Gram staining experiment, first, gentian violet was added for primary staining, and then iodine solution was added for counterstaining. Gram-negative bacteria, such as *E. coli*, *Salmonella*, *P. aeruginosa*, and so on, are becoming more and more resistant to commonly used antibiotics, partly because of the complex membrane structure. The structure consists of outer membrane and inner membrane, which forms cytoplasmic space. Toxic compounds can be absorbed by the cytoplasm and discharged directly from the body, thus reducing the number of drug molecules reaching the cytoplasmic target. The outer membrane of Gram-negative bacteria can effectively limit the active penetration of hydrophilic and hydrophobic molecules, which undoubtedly provides an additional protective factor. At the same time, both Gram-positive and Gram-negative pathogens were involved in multidrug resistance efflux pump. The multiple characteristics of efflux pump transporters lead to a common mechanism of drug resistance, that is, to enhance the role of antibiotic target mutation and other resistance mechanisms or promote the acquisition of drug modifications. The mutation of tumor suppressor genes is relatively random. Any position of the gene, regardless of any form of mutation, as long as the mutation causes the gene to lose its function, or its function is reduced, it may affect the occurrence of tumors.

In *E. coli* K12, the resistant tuberculosis differentiation (RND) efflux system includes acracarbtolc, acreacrfttolc, acraacrdtolc, mdtamdtb/mdtctolc, and yhiuyhiv TolC. *E. coli* is one of the most common bacteria in drug efflux pump. Generally, there are more than 30 kinds of jet pump. Among them, acrabtolc is the most important jet system. Acrabtolc system consists of three parts: outer membrane channel protein, membrane fusion protein (MFP) acra and efflux pump transporter acrB. Acra, acrB, and TolC play their respective roles in the acrabtolc jet system. When the expression of aclabtolc was the lowest, it was mainly regulated by acrR. At this time, if acrR does not exist, the acrbtolc system is regulated by the positive regulator Mara; soxs can activate the coding or operon of multiple resistance genes, such as aclab, TolC, MICF, and other genes activated by soxs, which can significantly enhance the drug resistance of *E. coli*. Different from Mara and soxs, rob has large molecular weight and exists in high concentration under normal conditions, which can ensure that it can completely penetrate the target promoter and regulate many genes including marRAB. MDR is unusual because it encodes three different transporters. TolC should be used as the outer membrane subunit of the drug efflux system dependent on the MFP, regardless of the type of endomembrane protein in *E. coli*. At the same time, the existence of Baer is not a necessary condition to ensure the complete activity of Baer overexpression in intact bacteria. The efflux system consists of outer membrane protein, additional protein, and internal and external transporters. Transporters located in the cytoplasm act as pumps, continuously discharging drugs, detergents, dyes, and other substrates. In clinical application, most efflux pumps of drug-resistant bacteria belong to RND family. Similar to fluoroquinolones resistance factors, a large number of Gram-negative bacilli were found before. Drug RND–MFP outer membrane factor (OMF) efflux pump system can adapt to a large number of unrelated chemical molecules, such as cationic antimicrobial peptides, fatty acids, bile salts, and sodium homoserine lactone. Carbapenems have become the first choice to treat ESBLs producing *E. coli*.

## 3. Experiment

### 3.1. Research Object

Enterobacteriaceae isolated from a hospital from January 2015 to June 2020 were selected.

### 3.2. Experimental Plan

Carbapenem susceptibility test and re-identification of drug-resistant strains: the sensitivity of Enterobacteriaceae to carbapenems was detected by microdilution method, and carbapenem-resistant strains were screened and identified by VITEK^®^2.

Resistance phenotype test: Detection of phenotype, modification test, IPM EDTA double disk collaborative test, IPM + EDTA composite disk test, ESBLs confirmation test, AmpC enzyme phenotype test, and sterility test: crude enzyme extract was seeded on Mueller–Hinton agar plate, incubated at 35°C overnight, and the next step was carried out for those without bacterial growth. If bacteria grow, follow-up experiments can be carried out after sterilization (centrifugation or repeated ultrasound).

MLST: The strains were sequenced, that is, 7 family genes (*rpoB*, *phoE*, *gapA*, *infB*, *mdh*, *tonB*, and *pgi*) of *K. pneumoniae* were amplified by PCR, and sequenced, compared with the database, and analyzed the sequence types of strains.

Drug sensitivity test: Etest paper was used to test the drug sensitivity of the original strain and the conjugate of subsequent transfer joint test. The operation steps are as follows: the bacteria are suspended in the incubator for 18–24 hours, the aseptic ring plate is carefully selected, the ground and bacterial suspension are evenly in normal saline, and the turbidity is adjusted to 0.5. Using sterile cotton, the bacterial suspension is immersed in the dense coated plate, and the surplus bacterial liquid is swabbed by rotating the cotton, and the bacterial suspension is extruded out of the inner wall of the test tube. After marking the agar plate with “cross,” draw it three times evenly. After each sealing coating, the plate was rotated 60° for the next dense coating to ensure the uniform distribution of the bacteria to be tested. Finally, a line is drawn along the inside edge of the plate. Open the plate cover, dry at room temperature, and paste Etest paper within 15 minutes. Use sterile tweezers to stick the Etest paper together, and use sterile tweezers to stick the drug-free end of Etest paper together, stick the minimum inhibitory concentration (MIC) value side up on the agar surface, and extrude the bubbles on the paper. In a large number of drug sensitivity tests, tweezers need to be disinfected in time. The paper cannot move after it is glued. Incubation record results: the drug sensitive plate was incubated in 35°C incubator for 16–18 hours. MIC values of various drugs were read according to the size of inhibition zone, and the results were recorded.

Conjugation test: The transferability of carbapenemase gene was detected by conjugation test. *E. coli* J53 (*E. coli* J53) is resistant to sodium azide and is a receptor strain. The single colonies of donor and recipient bacteria were added into 1 ml Luria-Bertani medium, respectively. Shake incubation at 35°C after 4 hours. The solution is based on the ratio of donor:recipient bacteria = 1:2 and incubation at 35°C for 4 hours.

The specific steps of enzyme-linked immunosorbent assay (ELISA) were as follows: coating antigen R1081-1-2 on 96 well plate, sealing with gelatin solution, incubating with antibody; after washing dishes, adding the second antibody labeled with peroxidase; adding tetramethylbenzidine phosphate buffer and hydrogen peroxide, and the reaction termination solution was sulfuric acid. The absorbance of the product was detected at 450 nm.

### 3.3. Experimental Results

According to the statistical analysis of the data, as shown in Figure 1 and Table 1, all strains were resistant to ceftazidime, ceftriaxone, ertapenem, and aztreonam. 87.5% of 14 strains were resistant to piperacillin. The results of drug sensitivity test showed that all strains were resistant to ceftazidime, ceftriaxone, ertapenem, and atranan.

According to the statistical analysis of data, as shown in Figure 2 and Table 2, MLST showed 5 carbapenem-resistant *K. pneumoniae* and 4 different types. The sequence types of kpn6099 and kpn6617 were the same.

According to the statistical analysis, as shown in Figure 3, kpn6617 is resistant to all *β*-lactamases and carbapenems, but sensitive to ciprofloxacin, polymyxin, and tigecycline. The sensitivity of *E. coli* J53 to aztreonam and tigecycline was higher than that of kpn6617. *E. coli* J53 was more sensitive to these two antibiotics, MIC values were 0.5 and 0.25 *μ*g/ml, respectively. In addition, the sensitivity of *E. coli* J53 to carbapenems was slightly higher than that of kpn6617.

According to the statistical analysis of data, as shown in Figure 4 and Table 3, PC is a positive control and NC is a negative control. The judgment criteria were the dilution value corresponding to OD450 value was greater than twice of NC, and more than 0.25 was the antibody titer. Therefore, the ELISA titer of the antibody was 1:40,000, and acrB antibody was successfully prepared.

### 3.4. Analysis and Discussion

Enterobacteriaceae, such as *E. coli*, *Klebsiella*, and Enterobacteriaceae are normal colonization bacteria and common opportunistic pathogens. The resistance of *E. coli* fertilized eggs to meropenem was higher, which may be due to more copies of drug-resistant genes in fertilized eggs. Kpc-2, IMPl–4 and NDM-1 are often multidrug-resistant or even total resistant, resistant to carbapenems, but sensitive to broad-spectrum lactams. The MIC of piperacillin and piperacillin/tazobactam for IMP4 producing transferred fertilized eggs was very low, while that of atrananine was low. EDTA can significantly reduce the MIC of carbapenems, which is consistent with the characteristics of metal caprolactam enzyme. Active efflux leads to drug resistance: drug efflux is an important mechanism of microbial resistance, which is completed by drug efflux pump (active efflux system). More precisely, the R family has four membrane transport regions: SMR/QAC (*Salmonella*), qacE (*Klebsiella* gas producing gene), and EmrE (*E. coli*). Some proteins of this family have oligomer functions. The RND series are usually used as a combination of three jet systems, which are more direct than the jet systems entering the peripheral plasma. *E. coli* acra, acrB, and tolcemra. TolC, MEXA, and mexb OprM are three jet systems, acrB and mexb are RND transporters, acra and MEXA are MFPs, and TolC and OprM are OMFs. Among them, MF, SMR, RND family use electrochemical H+ transmembrane gradient as the driving force, ABC family use ATP as energy source. LmrA (*Lactococcus lactis*) and MsrA (*Salmonella*) are transporters of chaperone family. Norm is part of the family. Norm is related to the active outflow of Na^+^. The detoxification process in detoxification system may be an extracellular process. Drug resistance of *E. coli* can be intrinsic or acquired through gene mutation and gene transfer.

Because ESBLs producing bacteria have multiple drug resistance, they are usually mediated by plasmid. Drug resistance can be transferred from one bacterium to another, or even between different strains. The risk factors for the prevalence of ESBLs are: application of arterial catheterization or central venous catheterization, recent surgery, especially acute abdominal surgery, gastric and duodenal catheterization, residence time, especially in ICU ward, birth weight below normal, use of antibiotics, previous home care, disease severity, catheterization, and assisted breathing. ESBL producing bacteria are usually resistant to a variety of antibiotics, including the third generation cephalosporins, quinolones, and aminoglycosides. Quinolone resistance genes are usually located on chromosomes. Quinolones resistance gene and ESBLs coding gene can be located on the same transferable plasmid. At the same time, the plasmids of ESBLs producing bacteria often carry chloramphenicol, sulfonamides, tetracycline, and aminoglycoside resistance genes. The resistance of ESBLs producing bacteria is related to plasmids carrying multiple drug resistance genes, ESBLs genotypes, and the inherent drug resistance mechanism of bacteria. It seriously affects the clinical anti-infective treatment through chromosomal changes or the transfer of drug-resistant plasmids and transposons.

## 4. Conclusion

(1) Kpn6617 was resistant to all *β*-lactamases and carbapenems, but sensitive to ciprofloxacin, polymyxin, and tigecycline. The sensitivity of *E. coli* J53 to aztreonam and tigecycline was higher than that of kpn6617. (2) Plasmid-mediated deletion of IMP-1 metallo-*β*-lactamase binding outer membrane protein is one of the main reasons for the decrease of antibiotic sensitivity. (3) The loss of outer membrane pore protein is also one of the common mechanisms of bacterial resistance. Compared with single antibiotic therapy, the combination therapy of multiple antibiotics has more obvious effect and can delay the generation of drug resistance.

## Figures and Tables

**Figure 1:** Drug sensitivity results.

**Figure 2:** Homology of strains.

**Figure 3:** Sensitivity comparison.

**Figure 4:** AcrB antibody titer.

**Table 1:** Drug sensitivity results.

Antibiotics	Drug resistance rate (%)	Intermediary rate (%)	Sensitivity rate (%)	MIC value
Piperacillin	87.5	12.5	0	40
Ceftazidime	100	0	0	56
Cefatriaxone	100	0	0	300
Aztreonam	100	0	0	100
Ertapenem	100	0	0	50

**Table 2:** Homology of strains.

Housekeeping genes	3059	5669	370	6099	6617
*rpoB*	1	1	1	37	37
*phoE*	1	1	13	93	93
*gapA*	1	3	2	18	18
*infB*	6	3	9	22	22
*mdh*	1	1	2	26	26
*tonB*	1	4	16	99	99
*pgi*	1	1	1	22	22

**Table 3:** AcrB antibody titer.

Antibody ID	6.25 K	12.5 K	25 K	50 K	PC	NC
R1081-1-1-2K1B1	3.186	2.931	2.599	1.966	3.173	0.119
R1081-1-1-2K1B1	2.741	2.174	1.52	0.958	2.967	0.109

## Data Availability

Data supporting this research article are available from the corresponding author or first author on reasonable request.
